# Community-Driven Family Planning in Urban Slums: Results from Rawalpindi, Pakistan

**DOI:** 10.1155/2023/2587780

**Published:** 2023-02-06

**Authors:** Adnan Ahmad Khan, Taimoor Ahmad, Areesha Najam, Ayesha Khan

**Affiliations:** ^1^Research and Development Solutions (RADS), Islamabad, Pakistan; ^2^Akhter Hameed Khan Foundation (AHKF), Islamabad, Pakistan

## Abstract

**Background:**

Pakistan's contraceptive prevalence rate (CPR) has remained static (less than 1% annual increase since 2006) due to several demand and supply issues. The Akhter Hameed Khan Foundation implemented a community-driven, demand-generation intervention with complementary supply side family planning (FP) services in a large urban informal settlement in Rawalpindi, Pakistan.

**Methods:**

The intervention recruited local women as outreach workers called Aapis (sisters), who conducted household outreach and provided counseling, contraceptives, and referrals. Program data were used to guide in-program corrections, identify the most willing to use married women of reproductive age (MWRA), and target specific geographic locations. The evaluation compared results from two surveys. The baseline survey included 1485 MWRA while the endline included 1560 MWRA that were sampled using the same methodology. A logit model was used with survey weights and clustered standard errors, to estimate the odds of using a contraceptive method.

**Results:**

CPR in Dhok Hassu increased from 33% at the baseline to 44% at endline. Long-acting reversible contraceptives (LARCs) usage increased from 1% at baseline to 4% at endline. Increase in CPR is correlated with increasing number of children and education of MWRA and is the highest between the ages of 25 and 39 and for working women. Qualitative evaluation of the intervention provided lessons about in-program corrections using data and empowerment of the female outreach workers and MWRA.

**Conclusion:**

The *Aapis* Initiative is a unique community-based demand-supply side intervention that successfully increased modern contraceptive prevalence rate (mCPR) by economically engaging the women from within the community as outreach workers and enabling healthcare providers to establish a sustainable ecosystem for increasing knowledge and access to family planning services.

## 1. Introduction

Pakistan is the fifth most populous country in the world with a population of 220 million that is growing at 2.4% annually [1]. This is associated with one of the highest fertility rates in the region at 3.55 (regional fertility rate ranges from 2.05 to 2.25) and the lowest Human Development Index at 151, relative to its peers—India (113), Bangladesh (119), Iran (73), and Sri Lanka (66) [2]. A signatory of the FP2030 (formerly known as FP2020), Pakistan, has struggled to meet its commitment to increasing its contraceptive prevalence rate (CPR) to 50% by 2025 and 60% by 2030. CPR in Pakistan has hovered around 35% since 2012, despite the considerable funding and programming by the government and donors [3].

Much of the programming in Pakistan has been supply side and rural [4]. The failure to increase CPR is often ascribed to a lack of awareness by end-users, inadequate engagement of men in the FP dialogue, missed opportunities of postpartum FP, and limited scale “project-driven” programming that are too small to have population level impact [4–6]. By contrast, nearly all successful interventions in Pakistan have ensured continuity of services or commodities and reached their beneficiaries through household outreach. Another key feature of all successful interventions is that they operated in large enough geographic areas, i.e., they reached a large enough population, where their impact could be measured. This contrasts with a number of interventions that showed some programmatic success but their impact was not measurable on national or subnational surveys [4].

In Pakistan, an important unexplored population is that of the urban poor. Approximately 30% of the population of Pakistan lives in informal urban settlements (slums) [6]. Many of these localities and their residents are undocumented and therefore excluded from public sector services. This reflects in the relatively low CPR (27%) and mCPR (24%) among the urban poor [3]. On the other hand, their physical presence in cities and their density make it much easier and cheaper to provide effective family planning (or other health) services in these communities.

MWRAs often opt for LARCs and continue it for a minimum of seven months when services are provided for free (vouchers) [7]. Voucher scheme is an effective intervention but this is often short term as it is funded externally. Therefore, it is not sustainable for making a lasting effect [8]. On the other hand, social franchising models have also contributed to increase uptake of FP services; however, private clinics are skeptical of locating in urban slums/rural communities as they seek to maximize their profit [9].

Community-based intervention is a hybrid model as it addresses both demand and supply side components of FP. In Malawi, a community-based model increased the contraceptive uptake for married women by 8.2 percentage point [10]. The effect was greater for women residing in rural communities with lower level of education and income, while Nigeria and Ethiopia have also increased contraceptive use by 22% and 390%, respectively, via community-based interventions [11, 12]. It has proven to be successful in many low- and middle-income countries because it provides service at the door steps; hence, it reduces social barriers, eliminates travel cost, provides access to contraceptives with referrals to nearby health care providers, and creates knowledge regarding FP.

The Akhter Hameed Khan Foundation (AHKF, formerly, the Akhter Hameed Khan Resource Center, AHKRC) was built on successful rural (HANDS Marvi) and urban (Sukh, Karachi) models from Pakistan to develop a community-based program to reach approximately 278,000 residents of Dhok Hassu, an urban slum in the heart of Rawalpindi, Pakistan, that spans over 4 union councils. Outreach workers were hired to provide door to door service to MWRAs in Dhok Hassu including counselling related to family planning, providing contraceptives (pills and condoms) and referrals to health care providers (HCP), hence addressing both demand and supply side issues for contraceptive use. The aim of this paper is to evaluate the effectiveness of this program to increase CPR and uptake of LARCs. We used a multimethod evaluation methodology using survey and program data to describe change in CPR and LARCs due to this intervention and the processes that may have contributed to this change.

## 2. Methods

### 2.1. The Population and Neighborhood

From January 2018 to April 2019 (16 months), AHKF implemented a community-based health and economic project in Dhok Hassu, Rawalpindi. The economic condition of the selected location ranges from very poor to lower middle class. Primarily, the main earners of households are associated with daily labor/wage earners. Spread over 1.84 km^2^ with a population of approximately 278,000, this area is classified by the city administration as poor/ultrapoor or an urban slum (UC 4, 5, 6, and 8, across 16 *Mohallah* or neighborhoods). The median household spending is PKR 32,000 (USD 288, in 2019 currency exchange rate of 1 USD = 111 PKR) a month, with a range of USD 47 to 497, as compared to national median of USD 273 and urban median of USD 297 [13].

### 2.2. The Intervention

36 outreach workers (called Aapis or sisters) were recruited from within the community to provide door-to-door counselling for family planning (FP), Business in a Box (BiB) products, contraceptives, and referrals. The selection was based on self-enrolment, time availability, and permissions from the household head to work outside the home. Selected Aapis received a 3-week interactive, pictorial-based, and low literacy-centered entrepreneurship training for counseling, marketing, sales, and basics of business management and planning, to enable local women as microentrepreneurs selling common need products to help community women overcome the issues of “mobility” and travel costs.

Aapis received a monthly stipend of PKR 3,000 (USD 27) and were asked to work for a minimum of 4-5 hours a day, 6 days a week, although work hours were not strictly monitored. Their income was further supplemented by a BiB revolving credit that was seeded with a grant of PKR 10,000 (USD 90) from which they could purchase common household or women-needed sale items such as sanitary pads, undergarments, cosmetics, baby diapers, kitchen supplies, and phone sim cards. Aapis had the flexibility to determine the products they carried and the pricing at which to sell them.

Aapis systematically visited and registered 35,771 households in the area, reaching 42,000 married women of reproductive age (aged 18-49 years) (MWRA). They used a one-page questionnaire to collect data on household demographics, FP needs, and empowerment indicators, provided FP counseling and contraceptives (condoms and pills), and referred women to local public or private clinics for long term contraceptive services (injections, IUCD, implants, or tubal ligation). Contraceptives were provided free of cost by the government's Population Welfare Department (PWD) and passed on to MWRA at no cost. Counseling technique was based on cognitive behavioral therapy (mCBT) that was adapted for low literate outreach workers in collaboration with the Department of Behavioral Sciences of the National University of Science and Technology (NUST), Islamabad.

Referrals were made initially to the local public sector clinic. From the third month onwards, referrals were expanded to 9 private providers (mainly female) that were trained by PWD trainers on family planning and LARCs, counseling and side effect management as part of a certified *Hamari Sehat* (our health) Network, and who carried a variety of method mix options. Healthcare providers (HCPs) also participated in the health camps and provided MWRA with antenatal or postnatal care along with FP services. They received supplies at subsidized costs (25% below market) that were replenished by AHKF.

If a MWRA accepted a new method or referral, *Aapis* would follow up on her in one week to ask about and provide support in case she encountered a side effect. Follow-up visits were based on a decision algorithm and recorded in the database.

A cluster of 6 Aapis was complemented with 1 male mobilizer. Male mobilizers (i) counseled spouses of MWRA that reported resistance to FP by their husbands (these were identified by the Aapis) and (ii) engaged local men in unstructured health-livelihood relevant discussions on economic benefits of smaller families and how they could expand income generation sources.

All data were recorded centrally, and key indicators such as number of visits by neighborhood, new users, and individual methods were depicted on an online dashboard. The project team reviewed this weekly with the research partner (Research and Development Solutions—RADS) to allow for program decisions.

### 2.3. Measurement Design

The project was monitored by comparing annual surveys of the location, along with in-program monitoring data. The annual surveys have been set up by RADS as part of its urban laboratory initiative and are extraneous to the current intervention. They used a multistaged clustered sampling approach. Using a UNICEF MICS 3 sample size calculator, and assuming a design effect of 2.5, a CPR of 35% with a marginal error of 95% confidence interval at 0.12, and allowing for up to 9% refusals, a sample size of at least 1,351 was chosen. This was rounded up to allow 5 respondents from each of the 300 clusters and a minimum of 50 respondents from each of the 17 neighborhoods.

A total of 1045 clusters were identified using Google Maps, and among these, 300 were randomly identified. 1,485 interviews were conducted at the baseline (November 2017) and 1,560 at the endline (January 2019). In each cluster, an origin point was ascertained randomly, and from that, every third household was included for survey. In case of nonresponse/refusals, the adjacent household was approached, and the sampling frame then shifted accordingly. Both baseline and endline surveys used the same sampling approach each time but not necessarily the same respondents. Refusals were less than 3%.

All respondents provided informed consent. Survey design, including consent, was approved by RADS IRB that is registered with the US NIH. It is important to note that surveys were not donor-funded but were part of our annual survey series that is supported through internal funding. Their internal periodicity required the endline to be conducted 3 months before the end of the project.

In addition to the surveys, program data were collected from Aapis' initial and follow-up household visits, from the commodity supplies and referrals. A total of 35,771 households (out of the estimated 40,000) were registered during the program. A one-page enrolment form asked about the number of children, current pregnancy, the respondent (MWRA) aspirations for family size, fertility choices, and intentions for FP use. A simpler follow-up form asked about any changes in family, method continuation, and any changes in use of or aspirations for FP. These data were collated on a dashboard that was displayed online for the team. The team reviewed these data weekly to inform programming decisions that included approaching women to start or switch methods (for example, to ask previous short-term method users for the option to switch to LARCs), identifying which *mohallas* or women needed more attention and followed overall trends of specific methods and any other emerging patterns.

### 2.4. Model Specifications and Data Sources

Our analysis uses annual surveys to estimate the odds ratios for the use of contraceptives and the use of LARCs among MWRA using separate logit models with probability weights and clustering standard errors on *mohallah* level. Since our dependent variables (CPR and LARCs) are binary, we opted for logistic rather than linear probability model (LPM).

We did not use LPM regression because outcome variables are binary; hence, they do not follow normal distribution which is essential for inference. Furthermore, standard errors are not correct under LPM, and probabilities are not restricted between 0 and 1. Moreover, the variance of binary variable always depend on values of covariates so there is always heteroskedasticity. Lastly, when the dependent variable is binary, the distribution becomes nonlinear due to which logistic regression is the appropriate method as it covers this aspect.

We have estimated a logistic regression model (regression 1) in which we are interested in the association of the visit of Aapi with the current use of contraceptive (*Y*_*it*_). The model specification is as below:

(1) $$\begin{array}{c} Y_{it}=\beta_{0}+\beta_{1}\text{ endlin}{\text{e}}_{\text{t}}+\beta_{2}\text{ Aapi Visi}{\text{t}}_{i}+\beta_{3}\text{ ag}{\text{e}}_{it}+\beta_{4}\text{childre}{\text{n}}_{it}+\beta_{5}{\text{education}}_{it}+\beta_{6}{\text{working}}_{it}+\beta_{7}\;{\text{sanitation}}_{it}+\beta_{8}\;{\text{rooms}}_{it}+\epsilon_{it}. \end{array}$$

Our main dependent variable, *Y*_*it*_, is a dichotomous variable which indicates the current use of any contraceptive method (current user = 1, 0 = otherwise) for a MWRA *i* at time *t* (*t* = 0 for baseline, *t* = 1 for endline). The main independent variable is the endline variable which takes the value 1 if the HH was surveyed in the endline and 0 if the HH was surveyed in baseline. To isolate the effect of the Aapi on the use of contraceptives, a binary variable, Aapi visit is defined, which takes the value 1 if the respondent recalls being visited by the Aapi and 0 otherwise (Table 1).

The regression also controls for other factors that correlate with the use of contraceptives. These include age, number of children of MWRA, education of MWRA, and whether a MWRA is currently part of the workforce. Household (HH) characteristics act as a proxy for the HH poverty levels—these include sanitation facilities and number of rooms.

The variable age takes the value 1 if a MWRA is aged between 25 and 35 and 0 otherwise; children, a categorical variable, takes the value 0 if MWRA has no children, 1 if MWRA has up to three children, and 2 if MWRA has more than three children. Education is categorized into 3 groups: 0 for less than primary education, 1 for up to primary or middle school, and 2 for matric and above. Working is a binary variable indicates if the women is currently working or not (working = 1, otherwise = 0). Sanitation is also a binary variable indicating the presence of improved sanitation facilities. Rooms signifies the number of rooms in the house and takes a value of 1 if there are three or more rooms in a household and 0 otherwise.

We have also included a second model (regression 2) to estimate the use of long-acting reversible contraceptives—LARCs for a MWRA *i* at time *t* (*t* = 0 for baseline, *t* = 1 for endline). The model specification is same as regression 1 but the dependent variable is LARCs which is given a value of 1 if the MWRA is a LARC user and 0 otherwise.

We performed postestimation diagnostic tests to check the assumptions for the multiple logistic regressions. We calculated mean variance inflation factor (VIF) to check the multicollinearity between independent variables, “lfit” command to investigate goodness of fit of the models, and lastly, likelihood ratio test (LR test) to check for the model specification (restricted vs. unrestricted).

## 3. Results

The median age of the MWRA is around 32 years. Around 62% at baseline and 70% at endline of the respondents were between the ages of 25 and39, 58% and 47% had no education, and only 5% and 9% are part of the labor force, at the baseline and endline, respectively (Table 2). At the baseline, 83% MWRA could recall being visited by an Aapi, while at the endline, only 50% remembered such a visit.

CPR in Dhok Hassu increased from 33% at baseline to 44% at endline. Main increase was in the uptake of LARCs (from 1% at baseline to 4% at endline), implants (0% to 2%), and traditional methods (from 1% to 8%) (Table 3).

The adjusted odds of using a contraceptive are 1.43 times higher for MWRA aged between 25 and 35 relative to all other age groups and increase with the number of children, increasing education of the MWRA, if the MWRA works and if their home has access to modern sanitation. We found no effect of Aapi visits and increasing size of residential dwelling (surrogate for wealth) on CPR (Table 4).

Adjusted odds of using LARCs increased by 3.44 times overall from baseline to the endline. Likelihood of using LARCs increases by 1.71 times if Aapi had visited a household and increases with increasing children. The adjusted odds of using LARCs are 2.38 times higher for MWRA aged between 25 and 35 relative to other age groups. These odds increase with increasing education and more than double if the MWRA is educated from primary to matric (grade 10) and intermediate (grade 12) or higher levels. We found no effect of MWRA's work, access to sanitation, and size of the home on the use of LARC.

The significance of the LR test indicates that unrestricted (multivariate regression) model is preferred as compared to the restricted model (univariate regression). There is no problem of multicollinearity between the independent variables as the mean VIF is small. The goodness-of-fit test indicates that the models fit the data well as the *p* value is higher than 0.05.

### 3.1. Program Data

Program data were collected from 35,771 household registrations and 25,467 follow-up visits. Over the course of the intervention, contraceptive use increased from 38% to 59%, corresponding to 7,688 additional users. AHKF supported 5,916 of these new users to start contraception while continuing support for 14,175 existing users with contraceptives or services. A clear shift was visible from short- to long-term and reversible methods in the program data as shown in Table 3 for the survey data. Overall, 23% of those that were either using a short-term method at the outset or had initially started with one during the project shifted to a LARC or injection. There was a 3% increase in implants and 5% in IUD. 1,731 users converted from short-term methods to LARCs, so that a total of 2,341 LARC users were added (30% contribution to method mix) by the project end (Figure 1).

#### 3.1.1. Conservative Norms and Role Models

The Dhok Hassu community has an ethnic mix of Punjabis (52%) and Pashtuns/Afghans (48%), with the latter having more conservative social norms. While intermingling and urbanization have challenged rigid ethnic norms, there are still stark differences in how the communities perceive FP outreach. Working in such an environment required the Aapis and the project team to be sensitive to social, ethnic, and religious sensitivities and collaborate widely with local CBOs and opinion leaders. Community women—particularly young women—felt motivated by Aapis as role models as with the passage of time women started approaching the center to become “Aapis.”

#### 3.1.2. Qualitative Assessment of the Model

A total of 11,413 counseling sessions (using a simplified/modified cognitive behavioral therapy—mCBT—approach that was tailored for low literate Aapis) were conducted with non-FP users. On monitoring, many of the sessions did not follow the intended mCBT protocols in that the sessions were quick and Aapis were judgmental and mainly intent on informing rather than listening and interacting with the clients. Some remedial training was done with limited improvements. However, despite this limitation, an additional 20% nonusers converted to FP use following counseling sessions (discussed in Discussion).

#### 3.1.3. Aapis BiB

Business in a Box (BiB) by Aapis was a major sustainability measure for the project. Aapis income (profits) from BiB increased over time to an average of PKR 4,000 a month (USD 30). There were 7 Aapis (19%) that were remarkably successful (over PKR 10,000 a month) in the BiB, while a third of Aapis were not able to sell very much at all (Figure 2). On the other hand, some that sold well were not very effective in counseling for FP and vice and versa.

#### 3.1.4. Aapis Performance and Attrition

A total of 65 Aapis were hired throughout the project, and 36 were retained at any given time. Initially, the attrition rate was a major challenge (>20%) which eventually settled to less than 10% after 5-6 months of project implementation through capacity building, gaining of community acceptance and awareness of the Aapis presence, and BiB income generation incentives.

Low literate Aapis initially struggled with the HH forms and BiB inventory and would often resign or stop showing up rather than “voice” the difficulties that they faced. It took the Aapis and the project team several months to understand the concepts of the FP model and the expectations of work. Slowly, over time (through repeated small group refreshers by the project team), a performance criterion was jointly developed, and Aapis were given weekly feedback on their HH visits and BiB inventory management. Their performance rapport with the community and counseling skills improved with the duration of their work. On average, each Aapi conducted 1,669 visits (including both household and follow-ups) during the roughly 14 months of the implementation period.

#### 3.1.5. BiB Reluctance and Learning

Aapis are low-literate local women with limited knowledge of financial management and lower still for a computerized or tablet-based inventory management system that the BiB aspect required. Most had never worked before. They viewed the monthly stipend as more income than they had earned previously, and many were not motivated for additional income from BiB. On the other hand, a few Aapis excelled in BiB sales but were not interested in counseling for FP. Some were successful enough to leave the program venture out on their own. Repeated refresher sessions on inventory reporting and management and communication skills were conducted throughout the project.

Beyond FP, Aapis had wider social impact within the community. Although AHKF had struggled to recruit Aapis initially, there were several spontaneous applications by local women to join as Aapis from 3-4 months into the project, usually from streets where Aapis lived. In informal discussions, Aapis and project personnel reported that women felt more empowered to step out of their homes.

### 3.2. Male Mobilizers

Six male mobilizers were engaged from local community. While the mobilizers were able to engage nearly 4,500 men/husbands, their experience highlighted several design issues. Male mobilizers were even more reluctant than the Aapis to *counsel* newly married/younger couples. Additionally, men in urban slums work 1-2 jobs and were not available during (daytime) working hours. When they were available, they were not very interested in family planning. Monitoring observations from the project suggests that men may engage with different entry points than women. The most promising entry points for men were income generation, employment, and local municipal issues. Any discussions of FP had to be embedded in these conversations and supplemented with private direct or phone counseling to those that expressed interest.

We had originally planned to also use aspects of positive deviance inquiry to drive FP demand among men. However, for most parts, this did not work since most men were either engaged directly or, when in groups, the main discussion remained on other topics. The inability to fully guide these discussions was related to skills of male mobilizers. For most part, these men had not worked previously in community mobilization.

### 3.3. Private Healthcare Providers (HCPs)

Nine private health care providers were trained as part of the *Hamari Sehat (Our Health) Network.* Of these, two started providing implant services at their clinics. HCPs also participated in the monthly health camps and provided MWRA with antenatal or postnatal care along with other non-FP services. Their quality of FP services was certified including upskilling in infection control and assuring supplies.

Aapis would refer MWRA for LARCs or injections for a nominal (5%) referral fee. The increasing number of referrals (i) helped improve these health care facilities as they saw their income rise (AHKF did not pay the providers), (ii) AHKF quality check supervisor guided HCPs in improving and addressing their quality and infection control gaps and provided IEC materials, (iii) supplied contraceptives at a 25% subsidy, and (iv) connected them to the local government (PWD) clinic for long-term sustainability.

On average, Aapis helped increase HCP clientele by 15-20 FP and >30 non-FP clients per month, increases of 25% and 40%, respectively, compared to their volumes prior to engagement with the program. This allowed for a sustainable increase in the uptake of FP through demand generation as complemented with a sustainable health care network, creating an ecosystem wide change. However, during the intervention, a large international donor agency started funding free IUCD and injections to the local HCPs, who then became unwilling to “purchase” the subsidized products from AHKF. To some extent the project was able to negotiate with the HCPs (long-term continuity vs. short free supplies).

#### 3.3.1. Ensuring Commodities

Throughout the project, commodities and services were consistently supplied by the Punjab Population Welfare Department (PWD). This included condoms and pills that the Aapis carried and injections or IUCD that were provided by PWD clinic in the neighborhood to which Aapis referred clients.

### 3.4. Program Costs

The programmatic costs were calculated for reaching 35,771 households, adding 7,688 additional users while serving the existing 14,175. The cost of reaching (outreach) each household was PKR 447 (USD 4.02), while services cost PKR 1105 (USD 9.95) per user served, or PKR 578 (USD 5.21) per CYP, excluding commodity costs.

## 4. Discussion

We describe results of a low-cost, community-based intervention that helped increase CPR by 11% in 15 months and enhanced the use of LARCS by 3% points in a poor urban community from Rawalpindi (Pakistan). Beyond the change in contraceptive uptake, there are lessons in what works in such a community (simple community-driven outreach, ensuring commodities, program tracking using a combination of paper and digital records, and in-program adjustments based on data), what may be difficult (sophisticated counseling through low literate female or male outreach workers at mass scale), and what may have to be better worked out (reaching and engaging men).

Our project was a major departure from mainstream development and health programs in Pakistan that have focused on rural areas. Conceptually, all components of our programming drew upon previous works that demonstrate high FP uptake through community-based outreach and distribution programs in low literate and poor women/couples [14–17]. For example, a combination of communication, community engagement, outreach, and facility support led to an increase in CPR by 7% overall and by 10% for the poorest two quintiles in six cities in India [17]. A similar set of services helped increase CPR by 10-12% in major cities of Kenya, Nigeria, and Senegal [18]. Similarly, in Pakistan, the Marvi project in rural Sindh and Sukh project in urban Karachi both resulted in 15-25% increase in CPR through dedicated outreach, ensuring supplies and other elements of care. However, with the exception of the Sukh project, almost all programming has been rural. Prior to our intervention, it has been unclear to what extent can outreach be done in urban areas that have different social norms, and the extent that costs can be kept low in cities where outreach workers may have other employment options. In Pakistan, urban outreach has been difficult and expensive, as most programs sought to replicate the very expensive lady health workers program by the government.

Globally and in Asia, urbanization has been a major driver of poverty reduction [19–22], by interlinking population density and “agglomeration” (bringing together of diverse skills and resources in close proximity) to create opportunities for the many [23, 24]. In our context, this means that many of the unserved women and couples live very close to where services are administered from but are not reached with services as their communities are under or nondocumented and therefore ignored by public administrators. In Dhok Hassu, there is only one population welfare clinic and one government dispensary for a population of 278,000.

Another factor in low FP use is low labor force participation for women in Pakistan (21.5%) is among the lowest among comparable nations and lower still in cities (9.5%) [25], when female employment is well correlated with lower fertility [26, 27]. Low labor force participation of women is also intertwined with low mobility of urban women, for example, in the RADS annual survey 2017, only 27% said they felt comfortable buying groceries from a corner store in their street without permission or chaperone. In this milieu, having an outreach worker bring information and commodities to the doorstep and accompany MWRA to the clinic can substantially change FP use. For Aapis, population density translates into shorter travel distances between clients and a larger client base for their business in a box. Collectively, these factors lead to more visits and lower costs of engagement.

Beyond direct benefits for FP, Aapis fostered a wider social dialogue about women's mobility outside their homes and working. Both are very low in Pakistani cities, including Rawalpindi. While 36 Aapis are not sufficient to substantially change such norms, at least they initiated a debate in the community and provided role models to their neighbors. For this to scale, initiatives like this must be backed with increased opportunities for women to engage in employment and income generation, perhaps in stages that start with work that is more culturally acceptable, such as that which can be done at and from home, and then scale it to more remote work.

Our intent was and remained in engaging women with little or no prior work experience as outreach workers, in order to create role models of empowerment and mobility within the community. While this was successful in both drawing out previously nonworking women—both directly and indirectly as other local women saw them as role models—into employment where they chose their own hours, it also created some recruitment issues. Essentially, these women were low literate, with reservations about visiting and engaging their neighbors for counseling or sales and, most profoundly, reluctance to offer FP services to young couples, etc. These required repeated training and value addressing sessions. They also needed multiple sessions on communication skills, as most were used to just “telling” their pitch and did not engage MWRA interactively. Similarly, male mobilizers were even more reluctant to talk about FP, and these difficulties were compounded when their target men were also reluctant. For both male mobilizers and Aapis, low literacy also led to many issues with data collection and record keeping.

A major component of success was the use of data and dashboard to use these data. Initially, very basic data were collected on paper form that were digitized into a database. Soon, it was recognized that this can become a census of all households, and these data were used to identify women with different needs. For example, if a MWRA accepted contraception for the first time and expressed comfort with condoms or pills, she was initiated on these. However, the data system then prompted the team to revisit this woman in 4 months to see if she felt comfortable in graduating to injections or LARC. Similarly, supervisors could see and direct Aapis to follow up within a week, any woman who was initiated on a new method. Field supervisors found it useful to run basic queries on data such as location of most visits, neighborhoods with most or least FP uptake, and distribution of methods by location very useful in planning their work.

The project cost USD 4.02 per household reached, USD 9.95 per user served, and USD 5.21 per CYP, all well below any comparable costs in the public sector Pakistan, including that for the lady health workers [4, 28], and much below regional costs [29, 30]. The program owes its low costs to working with the community women, many of whom were working for the first time. This may have added to the high turnover, as Aapis could leverage their newly acquired social skills and experience for better jobs elsewhere. On the other hand, the program ignited some mobility among previously inexperienced women. An additional factor was the high population density of an urban slum. Dhok Hassu has 278,000 residents living in 1.9 square kilometers, meaning that no location was more than 30 minutes by walking. Aapis could easily call upon all their clients, and their supervisors could fit in many monitoring or supervisory visits on site. A final factor was the support from the PWD that supplied all the contraceptives and most of the LARC services. Without these, per user costs may have been USD 1-3 higher.

Although only half the women recalled seeing an Aapi, MWRA had 1.03 times higher odds of using FP and 1.71 times higher odds of using a LARC if she remembered being visited by an Aapi. To our knowledge, there is no other household outreach in program areas, and Aapis were not pushed to promote either the brand Aapi or the organization. More importantly, even though sophisticated counseling using CBT as a base was designed, however, most Aapis did not have communication skills—and few learned—to administer it. A large increase in CPR despite this suggests the presence of a (initially unintended) “nudge” effect [31], in that, at least some women may have a latent need for FP but needed a nudge in the form of an Aapi asking them if they wanted to use FP. The program data showed, once they started, it was easy for a subset of these to graduate to more advanced methods as seen by the 23% of MWRA who shifted from short-term methods to IUCDs and/or injections. Change in CPR over time was the highest among those with no or low education, women aged 25-29 (a 14 percentage point increase from baseline to endline), women with 3 or more children (those with the most need, 16 percentage points), and 35 percentage points increase among the poorest households, exemplified as those with unimproved sanitation services.

For the 9 HCPs enrolled with the Hamari Sehat Network, the linkage helped increase client volumes by 25% for FP and 40% for non-FP services. Previous programs have shown similar increases in client volumes by linking outreach with providers [16]. In many discussions, public health experts have opined that adding FP services to a general service providers' repertoire may not be financially viable since quality FP services require longer visits than general medicine visits and are not necessarily better remunerated. Our findings complement previous work that adding outreach may render provision of FP services financially viable for private sector providers and may be a key step towards sustainable FP programming [16].

## 5. Limitations

The baseline survey was conducted in December 2017 (3 months before program deployment), while the endline was in August 2019, around 4 months before completion of project activities. This is because the funding of the two surveys came from different sources that required a slightly different schedule than the conventional pre- and postintervention surveys. This may mean that the effect of the programming was undermeasured by the endline survey.

Program data collection, management, and use was an evolutionary process. The organization had to develop protocols and had to revert to local and home-grown solutions including the development of the database and dashboard intramurally. There was a steep learning curve for all of these, as there was for getting the teams to start looking and using it in weekly program decisions. Addition of a research partner, RADS, helped the implementation team as a dedicated research team could support with analysis and interpretation of findings.

## 6. Conclusion

As Pakistan endeavors to find lower cost solutions for its stagnant CPR, a focus on its rapidly urbanizing cities and attention to simple ground up programs such as the one we present would provide valuable insights into what works. We show that household outreach is affordable, for government or donors, and economically empowers women. However, important unknowns such as correlates of demand in urban communities and sustainability of FP use by families and couples need to be studied further in different contexts.

## Figures and Tables

**Figure 1:** Long- and short-term method users added each month.

**Figure 2:** Monthwise sales and revenue.

**Table 1:** Summary statistics of variables.

Variable	Observation	Mean	Standard deviation	Min	Max
CPR	3,045	0.32	0.46	0	1
LARCs	3,045	0.02	0.15	0	1
Endline	3,045	0.51	0.50	0	1
Aapi visit	3,045	0.70	0.46	0	1
Age	3,045	0.61	0.49	0	1
Children	3,045	1.25	0.70	0	2
Education	3,045	0.80	0.80	0	2
Currently working	3,045	0.10	0.30	0	1
Sanitation	3,045	0.62	0.49	0	1
Rooms	3,045	0.54	0.50	0	1

**Table 2:** Demographic breakdown of MWRA across baseline and endline (%).

Characteristics	Baseline (%)	Endline (%)
Survey sample	1,485	1,560
Age		
<25	20	14
25-39	62	70
>39	18	16
Education^∗^		
No education	58	47
Primary–middle	34	23
Matric or higher	8	30
Working women^∗^		
No	95	91
Yes	5	9
Children		
No child	4	6
Up to 3	47	49
More than 3	49	45
Aapi visit^∗^		
No	17	43
Yes	83	50
Do not know	0	7
Rooms^∗^		
<3	55	42
≥3	45	58
Sanitation^∗^		
No	34	19
Yes	66	81

^∗^Statistically significant at the 95% confidence interval.

**Table 3:** CPR and method mix change from the baseline to the endline.

CPR	Baseline	Endline
Overall CPR	33	44
Method mix		
Condoms	17	16
Pills	3	3
Injection	6	7
Female sterilization	4	6
LAM^∗^	0	1
LARCS^∗^	1	4
IUCD	1	2
Implant^∗^	0	2
Traditional^∗^	1	8

**Table 4:** Adjusted odds ratios, 95% CI, and *p* values for multivariate logistic regression analysis on the use of contraceptives in Dhok Hassu, Rawalpindi (*n* = 2,652).

Variables	CPR	LARCs
Constant	0.005^∗^ (0.000593-0.0424)	0.004^∗^ (0.00119-0.0139)
Endline	1.48 (0.972-2.240)	3.44^∗^ (1.042-11.35)
Aapi visit	1.03 (0.781-1.370)	1.71^∗^ (1.059-2.765)
Age (less than 25 or more than 35)		
25 to 35 years of age	1.43^∗^ (1.285-1.601)	2.38^∗^ (1.083-5.232)
Children	(Reference: no child)	(Reference: more than 3 child)
Up to 3 children	37.46^∗^ (4.551-308.4)	0.35^∗^ (0.224-0.556)
More than 3 children	57.42^∗^ (6.881-479.2)7	—
Education (less than primary)		
Primary to matric	1.65^∗^ (1.397-1.939)	2.60^∗^ (1.711-3.947)
Intermediate or higher	1.71^∗^ (1.264-2.302)	3.93^∗^ (2.328-6.645)
Currently working	1.48^∗^ (1.021-2.154)	1.93 (0.729-5.105)
Sanitation	1.69^∗^ (1.270-2.245)	0.83 (0.372-1.835)
Observations	2,652	2,516
LR test	(Prob > chi^2^) < 0.001	(Prob > chi^2^) < 0.001
Mean VIF	1.18	1.18
Goodness of fit	(Prob > chi^2^) = 0.1704	(Prob > chi^2^) = 0.0885

1. Number of rooms were insignificant for both regressions; therefore, it is not included in the table. 2. For LARCs, number of children does not contain any response for no child; hence, reference category is more than 3 children. Robust confidence interval in parentheses. ^∗^Significant at 95% CI or above.

## Data Availability

The dataset used in this study is available on request from the authors.
